# A Phlegm Stagnation Monitoring Based on VDS Algorithm

**DOI:** 10.1155/2020/8714070

**Published:** 2020-01-24

**Authors:** Zhiguo Gao, Xin Yu

**Affiliations:** ^1^School of Artificial Intelligence and Information Technology, Nanjing University of Chinese Medicine, Nanjing 210044, China; ^2^College of Computer and Software, Nanjing University of Information Science and Technology, Nanjing 210044, China

## Abstract

In the nonmedical sputum monitoring system, a practical solution for phlegm stagnation care of patients was proposed. Through the camera, the video images of patients' laryngeal area were obtained in real time. After processing and analysis on these video frame images, the throat movement area was found out. A three-frame differential method was used to detect the throat moving targets. Anomalies were identified according to the information of moving targets and the proposed algorithm. Warning on the abnormal situation can help nursing personnel to deal with sputum blocking problem more effectively. To monitor the patients' situation in real time, this paper proposed a VDS algorithm, which extracted the speed characteristics of moving objects and combined with the DTW algorithm and SVM algorithm for sequence image classification. Phlegm stagnation symptoms of patients were identified timely for further medical care. In order to evaluate the effectiveness, our method was compared with the DTW, SVM, CTM, and HMM methods. The experimental results showed that this method had a higher recognition rate and was more practical in a nonmedical monitoring system.

## 1. Introduction

Phlegm stagnation, airway obstruction with phlegm, and other respiratory problems may occur during the care of older or terminal patients, resulting in serious complications such as hypoxia, asphyxia, pulmonary infection, and respiratory failure [1, 2]. To deal with such problems in the use of remote healthcare systems, a monitoring system is necessary to monitor the physiological parameters of patients in real time.

The respiratory monitoring mainly focuses on parameters of the frequency, intensity, duration of coughs, etc., to provide an important clinical reference for disease diagnosis, treatment, and drug-efficacy evaluation. So far, the analysis and recognition of cough mainly refer to the speech recognition system and depend on neural networks, dynamic time warping (DTW), the hidden Markov model (HMM), the classification tree method (CTM), and the k-means algorithm [3–10]. For example, Kou et al. [4] detected cough signals in continuous speech streams by using the keyword recognition method in the HMM. Yin and Mo and Shin [5, 6] made cough recognition by introducing a DTW-based [11, 12] classification model. The Hull Automatic Cough Counter (HACC) achieved automatic cough recognition by establishing a classification model with a probabilistic neural network (PNN). Drugman et al. and Wang et al. [7, 13] distinguished cough sounds from environmental sounds by establishing a hybrid model with both a neural network and a hidden Markov model. Sun and Zhu [14] distinguished the two kinds of sounds by using the classification tree method (CTM). Meng et al. [15] reduced noise and expanded the characteristics of breathing sound by an integrated serial algorithm. Niu et al. [16] detects sputum by using image processing techniques. Heretofore, no research concerns about the physical change of the human body for the diagnosis and prediction in cough relative respiratory monitoring system. However, in a practical monitoring system of older or terminal patients, phlegm stagnation and airway obstruction with phlegm are rarely solved by cough recognition technology [17]. We still need manual work to diagnose these dangerous symptoms. There is a wide gap between the current health monitoring system and the practical nonmedical monitoring system of older or terminal patients.

Cough recognition and extraction system can recognize cough signals and display the severity of the coughs and the efficacy of the treatment, which is convenient for doctors to diagnose. During the care of older and terminal patients with the phlegm accumulation symptom, a practical method is needed to monitor the patients in real time and give an early warning so that the caregiver can help the patient expel phlegm in a timely manner. However, there is no detailed and effective method currently. Therefore, a new method based on image detection is proposed in this paper. Firstly, the computer collects the video images of the patient's throat by a camera, and then a category learning algorithm proposed in this paper is used to analyze these video images. Finally, the computer sends the analyzed results to the client in real time, which can timely provide the patient with moderate care and decrease the risk of accidental death.

## 2. Related Work

### 2.1. The DTW Method

DTW has good performance in template matching. It generally uses an action in the training set as a template and compares actions to be recognized with the template. The action closest to the template is viewed as the action of the template. In our experiment, the nearest neighbor algorithm is used and each action corresponds to multiple templates. A test action can be recognized if we can find a template closest to it.

The main limitation of DTW is that it requires the monotonous change of a sequence over time. In motion recognition, however, actions occur according to time order. Besides, DTW is believed to have nice results in the experiment for the following reasons. (1) It utilizes multiple templates and adopts the nearest neighbor method. (2) It well displays the similarity in shape. Though DTW is replaced by HMM in speech recognition, it still plays an important role in motion recognition.

Since motion features cannot be represented by a single image, it is necessary to recognize actions by a plurality of sequential images. In this paper, actions are recognized through a sequence of images. From the above, we know how to obtain the similarity in shape between two images. But it is still difficult to obtain the similarity between sequential images because other information about the sequence is unknown, for example, the length and starting position of the sequence and the interval between sequences.

An advanced DTW algorithm is adopted in this thesis for sequence comparison. DTW was originally applied to speech recognition [18] due to its capability of handling the problem of inconsistent speed. There exist similar problems in action sequences, such as fast or slow pace and sometimes acceleration in pace. All these problems can be well disposed with DTW. Our VDS algorithm enhances DTW with the combination of SVM for target classification, which will improve the accuracy of the recognition results.

Suppose there are two action sequences *x*_1_,…, *x*_*m*_ and *y*_1_,…, *y*_*n*_, where *M* and *N* represent the lengths of the two action sequences respectively, then the DTW distance *D* (*i*, *j*) of the two action sequences can be calculated with the following:

(1) $$\begin{array}{c} D\left(i,j\right)=\min\left\{D\left(i,j-1\right),D\left(i-1,j\right),D\left(i-1,j-1\right)\right\}+d\left(x_{i},y_{i}\right),\;i=1,\ldots ,M,j=1,\ldots ,N. \end{array}$$

The distance function *d*(*x*_*i*_, *y*_*i*_) is a matching distance of two motion sequences that is obtained with dynamic rules:

(2) $$\begin{array}{c} d\left(x_{i},x_{j}\right)=\frac{1}{n}\underset{p_{k}\in x_{i}\;q_{t}\in x_{j}}{\sum }\;\min c\left(p_{k},A\left(q_{t}\right)\right)+\frac{1}{m}\underset{p_{k}\in x_{i}\;q_{t}\in x_{j}}{\sum }\;\min c\left(p_{k},A\left(q_{t}\right)\right). \end{array}$$

From (*M*, *N*), we can find the matching path by roll back. When rolling back to (1,1), we will get the shortest path. The initial value of *D* (*i*, *j*) is 0 when *i* or *j* is less than 1.

Figure 1(a) shows the local path constraints of *D*(*i*, *j* − 1), *D*(*i* − 1, *j*), and *D*(*i* − 1, *j* − 1). They are the essential constraints during the matching of two action sequences.  Figure 1(b) is another local path constraint, corresponding to a new DTW value that should be recomputed in formula (1). The motion is generated in chronological order in motion recognition, and the shape is sequentially changed accordingly. Therefore, the path constraint [19] of Figure 1(a) can well describe the change of the motion sequence.

### 2.2. SVM Strategy

Next, we will use SVM to achieve action classification. Set the linear separable sample set *D*=(*x*_*i*_, *y*_*i*_), *i*=1,2,…, *l*, *x* ∈ *R*^*d*^, *y* ∈ {+1, −1} to be the category label. For linearly inseparable samples, a relaxation term *ξ*_*i*_ ≥ 0 is introduced. A general form of the linear discriminant function is *g*(*x*)=*w* · *x*+*b*, and the classification equation is (*w* · *x*)+*b*=0, which transforms the optimized hyperplane problem into convex quadratic programming:

(3) $$\begin{array}{c} \left\{\begin{array}{c} \Phi \left(w,\xi \right)=\frac{1}{2}w^{2}+C\left(\overset{l}{\underset{i=1}{\sum }}\xi_{i}\right),\\ \text{s}.\text{t}.\;y_{i}\left[\left(w\cdot x_{i}\right)+b\right]-1+\xi_{i}\geq 0, \end{array}\right. \end{array}$$

where *C* is the penalty factor. The constraint of formula (3) can be transformed into a maximization problem:

(4) $$\begin{array}{c} \Phi \left(w,\xi \right)=\frac{1}{2}w^{2}+C\left(\overset{l}{\underset{i=1}{\sum }}\xi_{i}\right)-\overset{l}{\underset{i=1}{\sum }}a_{i}\left\{y_{i}\left[\left(w\cdot x_{i}\right)+b\right]-1+\xi_{i}\right\}, \end{array}$$

where *a*_*i*_ > 0 is a Lagrangian coefficient. The optimal classification function is obtained by solving the Lagrangian function:

(5) $$\begin{array}{c} f\left(x\right)=\mathrm{sgn}\left\{\overset{l}{\underset{i=1}{\sum }}a_{i}^{*}y_{i}K\left(x_{i},x\right)+b^{*}\right\}, \end{array}$$

where sgn( ) is the symbol function; *l* is the number of training samples; *K*(*x*_*i*_, *x*) is the kernel function; *x*_*i*_ is the training sample; *x* is the sample to be decided, *b*^*∗*^ is the threshold determined by the training sample; and *a*_*i*_^*∗*^ is determined by the quadratic programming, and the kernel function is *K*(*x*, *y*)=exp(−((‖*x* − *y*‖^2^)/2*σ*^2^)).

Since SVM can only handle vectors with the same length, different sequences of eigenvectors cannot exist in the same vector space. Different length of motion sequence data will bring low resolution, and thus lead to less obvious separation effect. Our VDS model is capable of matching motion sequences automatically so that distances and similar velocity between motion sequences can reflect the similarity in symptoms, and thus achieve higher recognition accuracy of phlegm stagnation symptom accordingly. In VDS, the choice of kernel function will directly affect the accuracy and operation time. Considering the coincidence with DTW, we choose the radial basis kernel function. The inner product kernel function of RBF/VDS is obtained by combining the velocity characteristic parameters of sequential images:

(6) $$\begin{array}{c} K\left(x_{i},x\right)=\exp\left\{\frac{-{\left(\partial D+\left(1-\partial \right)V\right)}^{2}}{\sigma^{2}}\right\}, \end{array}$$

where *D* is calculated by the DTW, that is, *D* (*i*, *j*) in formula (1). The improvement of SVM kernel function will not affect the construction model and training of SVM, thus we can use SVM training method to make the classification of phlegm stagnation status [20].

## 3. Design of Phlegm Stagnation Learning Algorithm Based on Image Recognition

To judge whether the patient has phlegm stagnation symptom, this thesis proposes a Velocity Distance Support (VDS) algorithm. It processes the velocity of the moving target with the DTW algorithm and combines the classification of sequential images with the support vector machine (SVM) to identify the physical condition of the patient. The monitoring system sends the message back to the client in real time so that the caregiver can deal with problems promptly. The similarity distance between the feature vectors of input data and the prototype is calculated by DTW. It is a method based on nonparametric models. These methods can simply be implemented and can automatically match action sequences and calculate the distance between two sequences as well, while keeping a higher recognition rate than general methods based on parametric models. They can combine the similarity distance with velocity and then establish a laryngeal action identification model based on the SVM classifier. The diagnosis of phlegm stagnation can be carried out through parameters learning of the original training data set and classification of phlegm stagnation status.

### 3.1. Intelligent Video Surveillance System Structure

In a remote care system, the intelligent video monitoring system is introduced to help patients with phlegm accumulation. This intelligent video monitoring system can automatically record the video images of the scene monitored in real time through a camera. Then it will process and analyze these video frames to find the moving areas and extract moving targets from them [21], judge an abnormal phenomenon according to the relevant information of the moving target, and make an appropriate early warning for the abnormality. Thus, it can assist caregivers to deal with phlegm accumulation problems more effectively and make the care convenient. The process consists of video image input, moving target detection, feature extraction, classification training, warning module, etc. The overall process is shown in Figure 2.

### 3.2. Moving Target Detection in Video Images

With the rapid development of motion detection technology, more and more researches have been carried out for motion detection. There also exist great differences in the algorithms when targets have different shapes, detection environments, or camera properties changes. Most detection algorithms have some deficiencies and cannot provide satisfactory detection results. Motion detection algorithms mainly include interframe differencing, background subtraction, and the optical flow method [8]. Due to the complexity and heavy computation cost, the optical flow method has poor real time performance; thus, it generally needs independent hardware support [10, 11]. To avoid these problems, the intelligent video monitoring system for older or terminal patients described in this paper will turn to a three-frame differencing.

Interframe differencing is a time-based differencing algorithm. It is a technique where the difference between two neighboring video frames is checked and a differencing image is obtained. Then, the moving target is picked out from the differencing image after smoothing, binarization, and other processing. For each pixel in a frame, two consecutive frames are differenced by the following formula:

(7) $$\begin{array}{c} D\left(x,y\right)=\left|\;f_{k}\left(x,y\right)-f_{k-1}\left(x,y\right)\right|,\\ R\left(x,y\right)=\left\{\begin{array}{cc} 1, & D\left(x,y\right)\geq T,\\ 0, & D\left(x,y\right)<T, \end{array}\right. \end{array}$$

*f*_*k*−1_(*x*, *y*) represents the gray value of the pixel of the *k* − 1th frame, *f*_*k*_(*x*, *y*) represents that of the *k* th frame, *D*(*x*, *y*) represents the differential result, *R*(*x*, *y*) represents the binarization result, and *T* is the preset threshold. With too large *T*, there will be incomplete detection or leak detection; and on the contrary, there will be a lot of noise. The processing of interframe differencing is shown in Figure 3:

Generally, the detected moving target is regarded as the foreground image, and the other areas are background [12]. There is little difference between two consecutive frames in the value of background pixels or the difference only occurs in a very small area, but the pixels where the moving targets are located may change obviously. Therefore, a threshold filtering and morphological processing are carried out for the differential image. Finally a sufficiently large area with pixel changes is chosen as the moving target. This algorithm is simple and easy to implement, with adaptable and fast computational performance.

The results of interframe differencing are those areas with pixel changes in two consecutive frames. For areas with pixel changes in two consecutive frames where the moving targets are located, including the area where the moving targets were located in the previous frame and that in the current frame, the results are the sum of two areas with pixel changes. This means that the target displayed in the resulting image is larger than the actual one, which is called an image tail [13]. Besides, as many targets have little change in pixels by themselves, the areas with the moving targets in both frames also have little change in pixel values and are likely to be taken as foreground images. This appears as “holes” inside the detection results [14] and may weaken the detection effect of the interframe differencing largely.

To overcome the shortcomings of interframe differencing, a three-frame differencing was proposed. It extracts three consecutive frames (*k* − 1, *k*, and *k* + 1) and makes differencing computations on *k* − 1, *k* frames and *k* − 1, *k* frames, respectively. Then, an AND operation is performed on the differential images to remove the elongated portion of the moving target. Therefore, the moving target obtained by the three-frame differencing is more accurate than the interframe differencing, but there will still be some holes in the simultaneously detected moving target. The formula of three-frame differencing is described as follows:

(8) $$\begin{array}{c} D_{1}\left(x,y\right)=\left|f_{k}\left(x,y\right)-f_{k-1}\left(x,y\right)\right|,\\ D_{2}\left(x,y\right)=\left|f_{k+1}\left(x,y\right)-f_{k}\left(x,y\right)\right|, \end{array}$$

(9) $$\begin{array}{c} R_{1}\left(x,y\right)=\left\{\begin{array}{cc} 1, & D_{1}\left(x,y\right)\geq T,\\ 0, & D_{1}\left(x,y\right)<T, \end{array}\right.\\ R_{2}\left(x,y\right)=\left\{\begin{array}{cc} 1, & D_{2}\left(x,y\right)\geq T,\\ 0, & D_{2}\left(x,y\right)<T, \end{array}\right. \end{array}$$

(10) $$\begin{array}{c} R\left(x,y\right)=R_{1}\left(x,y\right)\wedge R_{2}\left(x,y\right). \end{array}$$

*R* (*x*, *y*) denotes the resulting moving target, and ∧ denotes an AND operation. Three-frame differencing is an improved version of interframe differencing. It solves the problem that the moving object is elongated and enlarged during the use of interframe differencing. When the target color is close to the background, there will be some omissions during detection, resulting in an incomplete moving target. The processing of three-frame differencing is shown in Figure 4.

### 3.3. Feature Parameters Extract from the Moving Target

Extracting feature parameters from the moving object means transforming abnormal and abstract behaviors into detailed digital features, and the velocity feature can also describe the behavioral features of the moving object. Velocity is a common physical quantity. In a short time, the velocity *v* can be calculated by the ratio of the displacement *s* of the moving object to the time interval *t*. It fulfills the relation *v*=*s*/*t*.

When velocity is used to describe the behavior of a moving target, it can be regarded as a point particle. In planar geometry, when a point particle moves from position *a* to position *b* through a certain period of time *t*_0_, the coordinates of the positions *a* and *b* are recorded as *a* (*x*_*a*_, *y*_*a*_) and *b* (*x*_*b*_, *y*_*b*_), respectively.

Formula (11) denotes the distance that a point particle moves within the time period *t*_0_.

(11) $$\begin{array}{c} d_{0}=\sqrt{{\left(x_{2}-x_{1}\right)}^{2}+{\left(y_{2}-y_{1}\right)}^{2}}. \end{array}$$

After calculation of the distance *d*_0_, the velocity *v*_0_ of the point particle in the given time period *t*_0_ can be calculated with *v*_0_=*d*_0_/*t*_0_.

Because the behaviors and actions of moving objects change with time, the features for extraction are also changing. When the object moves from one position to another, the coordinates of its mass center are also changing. Therefore, the displacement of an object over a period can be denoted by the changes in the coordinates of the mass center. Given the frame rate of a video object *f*_*w*_, the moving object in the video has coordinates of mass center *f*_1_ (*x*_1_, *y*_1_). After one frame of moving, the coordinates of the mass center change to *f*_2_ (*x*_2_, *y*_2_). The displacement of the moving object that occurred during the above process can be calculated by (12).

(12) $$\begin{array}{c} l=\sqrt{{\left(x_{2}-x_{1}\right)}^{2}+{\left(y_{2}-y_{1}\right)}^{2}}, \end{array}$$

and the time it used is *t*=1/*f*_*w*_

According to the velocity formula of moving objects, it is easy to obtain the velocity of a moving object between adjacent frames. In this way, the velocity features of the moving target can be extracted with *v*=*l*/*t*.

### 3.4. Combining DTW Algorithm and SVM Algorithm for Sequence Image Classification

After target detection, the SVM model should be trained. The input of the SVM classifier is the extracted sample features, and the output is the resulting classification decision {1, 1}. Generally, the value −1 means action does not belong to the class of phlegm stagnation while value +1 means the action belongs to this class [22]. The training process of the SVM classifier is described as follows:

 
*Step 1.* Prepare a training set. Divide the training set into the same number of male and female sample sets, which should include a positive sample set and a negative sample set. The size of the training sample set directly affects the classification performance of the SVM classifier. The larger the training sample set is, the better the classification performance will be, and the sample set should include all possible cases.
 
*Step 2*. Place the positive and negative samples in different folders and normalize the size of all training samples.
 
*Step 3*. Complete feature extraction of positive and negative samples and assign “+1” or “−1”olabels to all positive and negative samples, respectively.
 
*Step 4*. Input the positive and negative sample features and labels into the SVM for sample training and finally obtain the SVM target classifier.

Next is the target detection and recognition with VDS. First, carry out the feature extraction of targets to be detected. Work out the distance of two sequence images with DTW. Input velocity features into the trained SVM target classifier. Finally, the classifier will output class decisions. In this way, the target recognition process is accomplished.

## 4. Experiments and Result Discussion

The laryngeal video images were processed by three-frame differencing, and the effect was shown in Figure 5.  Figure 5(a) is the test images without a sticker.  Figure 5(b) is the detection image with a sticker. Figures 5(a)(a1)–5(a)(a10) are the originally collected video images without stickers and the results obtained by simulation. Figures 5(b)(b1)–5(b)(b10) are the originally collected video images with stickers and the simulation images. From these comparisons, we can see that images with stickers make the target clearer and easier to detect, which improves the accuracy in target feature detection and recognition. Therefore, this paper detected phlegm stagnation symptoms in patients with stickers in the throat to obtain better recognition accuracy. In practice, we can achieve the sticker effect by putting something on the patient's throat.

Samples used in the experiment were video images collected in those with the phlegm stagnation symptom from October 2017 to February 2018. On the MATLAB platform, the three-frame differencing method was implemented to extract moving objects from video images. The velocity of moving targets was extracted, and then the samples (i.e., the test set) were classified and recognized with the VDS algorithm. In this paper, we compared the VDS algorithm with DTW, SVM, CTM, and HMM algorithms in the target detection rate and average running time under the same sample size and different sample sizes. The selected sample size was 50, 100, 150, 200, 250, and 300 male samples and the same number of female samples. The male samples are divided into two categories, namely, phlegm samples and nonphlegm samples. Phlegm samples and nonphlegm samples were tested at 25, 50, 75, 100, 125, and 150. Female samples were tested in the same situation as male samples. The detection rate and average running time of phlegm and nonphlegm samples in male and female samples were shown in Figures 6–11 and Tables 1–3. According to Tables 1–3, the detection rate of male samples, including both phlegm and nonphlegm, is higher than the female sample detection rate; the average running time of the experiment is lower than the average running time of the female sample. This is because the male throat features are more prominent and thus easier to detect and identify. According to Figures 6–11, the detection rate and average running time of the algorithm proposed in this paper were both significantly better than the other four algorithms, which means our method owns significant advantages. The feature of the SVM, CTM, and HMM classifier is that the larger the sample set is, the better the classification performance it will have. So the trends of the VDS, SVM, CTM, and HMM algorithm curves were different from the DTW algorithm. The recognition time of DTW is proportional to the number of training samples, and the overall efficiency is very poor. Compared with the DTW model, the VDS, SVM, CTM, and HMM have very short training time and recognition time, which gives the VDS obvious efficiency advantages in the analysis of the monitoring results. Therefore, the combination of DTW and SVM algorithm can automatically match the action sequence, and the distance between the laryngeal action sequences and the similar rate can reflect the similarity of the symptoms, thus achieving a higher recognition rate of phlegm stagnation symptom. Experiments showed that the proposed method was applicable to the phlegm stagnation monitoring system. When the VDS algorithm recognized the phlegm stagnation symptom, the alarm device starts immediately. The caregiver can make timely sputum suction for patients. It can not only monitor the patient's physical condition in real time and thus promote the performance of the monitoring system but also brings more convenience to the caregiver. Free from real time manual monitoring, the caregiver is largely relaxed.

## 5. Conclusions

This paper proposed a VDS algorithm for phlegm stagnation symptom recognition in nonmedical sputum monitoring system. It combines speed characteristics, DTW, and SVM to identify laryngeal actions and classify phlegm stagnation status. The experiments showed that our method can adapt to the laryngeal movement of different lengths and speeds. It is applicable to the phlegm stagnation symptom identification and monitoring system. When the VDS algorithm recognizes the phlegm stagnation status, an alarm device is activated immediately. The nursing staff can solve the problem of phlegm stagnation easily by using the suction method, which can monitor the patient's condition in real time, improve the monitoring system, and bring great convenience to the nursing staff as well. With no need of manual operation all the time, our method will greatly reduce the pressure of nursing staff.

## Figures and Tables

**Figure 1:** Different path constraints. (a) Path constraint *a*. (b) Path constraint *b*.

**Figure 2:** Process of intelligent video surveillance system.

**Figure 3:** Process of interframe differencing.

**Figure 4:** Process of three-frame differencing.

**Figure 5:** Effect of three-frame differencing for laryngeal video images. (a) Detection without a sticker. (b) Detection with a sticker.

**Figure 6:** Detection rate of male phlegm samples.

**Figure 7:** Detection rate of female phlegm samples.

**Figure 8:** Detection rate of male nonphlegm sample.

**Figure 9:** Detection rate of female nonphlegm samples.

**Figure 10:** Average detection time on male samples.

**Figure 11:** Average detection time on female samples.

**Table 1:** Detection rate of phlegm samples (%).

	VDS (male)	VDS (female)	SVM (male)	SVM (female)	DTW (male)	DTW (female)	CTM (male)	CTM (female)	HMM (male)	HMM (female)
50	93.5	92.7	86.7	85.1	84.6	83.9	84.9	82.3	81.9	80.3
100	94	93	88	85.9	84	82.9	86.9	84.8	84.5	84.4
150	95.3	94.1	89.5	86.5	83.3	81.7	88.4	85.3	87.5	87.3
200	96.7	95.4	91	88	82.1	80.2	89.0	87.6	90.7	90.3
250	97.3	96.3	92.1	89.3	80.6	78.4	90.7	89.6	91.2	90.5
300	98.8	97.2	93.4	92.6	78.4	77.6	91.3	90.5	91.7	90.6

**Table 2:** Detection rate of nonphlegm samples (%).

	VDS (male)	VDS (female)	SVM (male)	SVM (female)	DTW (male)	DTW (female)	CTM (male)	CTM (female)	HMM (male)	HMM (female)
50	96.5	95	88.7	88.1	94.1	93.4	86.3	85.2	84.6	83.3
100	97	96.7	90	89	93	92.3	88.1	87.2	87.8	87.5
150	97.3	96.8	90.5	90	90.3	89	90.3	89.2	90.5	90.3
200	97.7	97.7	92	91.2	87.1	86.1	91.3	91.1	92.2	92.2
250	98.3	98	94.8	94.8	85.6	83.6	93.8	93.2	92.5	92.3
300	98.8	98.8	95.4	95.4	80.4	78.4	94.9	94.4	92.8	92.5

**Table 3:** Average detection time of samples (ms).

	VDS (male)	VDS (female)	SVM (male)	SVM (female)	DTW (male)	DTW (female	CTM (male)	CTM (female)	HMM (male)	HMM (female)
50	62	64	70	71	75	77	75	78	81	84
100	68	69	79	81	86	89	84	87	87	89
150	75	78	90	92	99	103	96	97	98	102
200	81	84	103	105	115	117	113	115	118	122
250	87	88	114	116	133	136	126	129	143	144
300	95	96	125	127	156	159	145	149	159	160

## Data Availability

The image data used to support the findings of this study are available from the corresponding author upon request.
